The article "Urease and α-Chymotrypsin Inhibitory Activities and Molecular Docking Studies of Alkaloids Isolated from Medicinal Plant Isatis minima Bunge" was published in 2022. Journal: Evid Based Complement Alternat Med.

# Urease and *α-*Chymotrypsin Inhibitory Activities and Molecular Docking Studies of Alkaloids Isolated from Medicinal Plant *Isatis minima* Bunge

**DOI:** 10.1155/2022/1904874

**Published:** 2022-06-15

**Authors:** Fozia Fozia, Ijaz Ahmad, Zia ul Haq, Abdul Wadood, Hidayat Ullah Khan, Mushtaq Ahmed, Nargis Jamila, Riaz Ullah, Amal Alotaibi, Mujeeb A. Sultan

**Affiliations:** ^1^Boichemistry Department, Khyber Medical University Institute of Medical Sciences, Kohat, Khyber Pakhtunkhwa, Pakistan; ^2^Department of Chemistry, Kohat University of Science & Technology, Kohat, Khyber Pakhtunkhwa, Pakistan; ^3^Institute of Public Health & Social Sciences, Khyber Medical University, Peshawar, Khyber Pakhtunkhwa, Pakistan; ^4^Department of Biochemistry, Abdul Wali Khan University Mardan, Khyber Pakhtunkhwa, Pakistan; ^5^Department of Chemistry, University of Science & Technology, Bannu, Khyber Pakhtunkhwa, Pakistan; ^6^Department of Biotechnology, University of Science & Technology, Bannu, Khyber Pakhtunkhwa, Pakistan; ^7^Department of Chemistry, Shaheed Benazir Bhutto Women University, Peshawar, Khyber Pakhtunkhwa, Pakistan; ^8^Department of Pharmacognosy (MAPPRC, College of Pharmacy, King Saud University, Riyadh, Saudi Arabia; ^9^Department of Basic Science, College of Medicine, Princess Nourah Bint Abdulrahman University, P. O. Box 84428, Riyadh 11671, Saudi Arabia; ^10^Department of Pharmacy, Faculty of Medical Sciences, Aljanad University for Science and Technology, Taiz, Yemen

## Abstract

Phytochemical studies on the alkaloids fraction of the entire plant of *Isatis minima* Bunge resulted in the alkaloids **1–4** isolation, which were first time isolated from this species. The 1D and 2D NMR spectroscopic data were used to identify their structures, and there was satisfactory compatibility of the data compared to those which were previously published. In the examined compounds **1–4**, Isaindigotidione (**3**) and Isaindigotone (**4**) were shown as an effective urease inhibitor in such a concentration-dependent way against Jack bean and *Bacillus pasteurii* urease, with IC_50_ values 29.03 ± 0.04, 20.04 ± 0.09 and 34.03 ± 0.07, 26.13 ± 0.08 *μ*M, respectively. Compounds **3** and **4** were likewise shown to be an effective inhibitor against *α*-chymotrypsin, exhibiting IC_50_ values 16.09 ± 0.07 and 22.01 ± 0.06 *μ*M, correspondingly. The program MOE-Dock was used to perform a molecular docking analysis to confirm probable binding modes of the active complexes of the isolated compounds **1–4** and the crystal structure of urease and *α*-chymotrypsin enzymes. Compound **3** was the most active, having the highest docking scores against *Bacillus pasteurii* urease, *α*-chymotrypsin, and Jack bean (−8.6876), (−7.6647), and (−13.1927) *μ*M, respectively. All four alkaloids (**1–4**) showed significant urease and protease inhibitory potential and further these activities were confirmed with the help of molecular docking study.

The article "Urease and α-Chymotrypsin Inhibitory Activities and Molecular Docking Studies of Alkaloids Isolated from Medicinal Plant Isatis minima Bunge" was published in 2022. Journal: Evid Based Complement Alternat Med.

## 1. Introduction

The plant genus *Isatis*, which belongs to the Brassicaseae family, encompasses 50 taxa that are mostly found in the Irano-Turanian area. It represents seven species, which are found in Pakistan [1]. A perennial plant species *Isatis tinctoria* has been used for the formation of blue dye indigo throughout the centuries and usually referred to as woad. Currently, woad is utilized in modern medicine and Chinese folk [2]. A conventional medicine of China is “Ban-LAN-Gen” that is frequently employed for anti-inflammatory, antiviral, detoxification, and antipyretic purposes. It was assumed that its original source was originated from the plant dehydrated (dried) roots, including *Strobilanthes cusia*, *Isatis tinctoria*, and *Isatis indigotica* [3, 4]. According to modern statewide research, the major components of “Ban-LAN-Gen” were determined from the *Isatis indigotica* roots and were documented as shown in Pharmacopoeia of China (1990 Edition) [5]. The genus *Isatis* was used for the investigation of *α*-chymotrypsin and urease components that is a part of ongoing research [6]. The ethnopharmacological significance of a said *Isatis* genus encourage us to explore the bioactive components of *Isatis minima* Bunge, that is found in Quetta, Baluchistan, Pakistan and locally used to treat viral infection through local practitioner (Hakeems). Our prior research is the oxindole alkaloids isolation from the *Isatis costata* plant species [7, 8]. Phytochemical investigation of the genus *Isatis* revealed the isolation and structure elucidation of indole alkaloids, quindoline alkaloid, quinoline alkaloids, quinazolinone alkaloids, simple amide alkaloid, monoterpenes, methyl 2-acetoamidobenzoate, *β*-sitosterol, and ursolic acid [7, 9, 10], while no phytochemicals are reported so far from *Isatis minima* Bunge species.

The ethanol soluble fraction of the *Isatis minima* Bunge plant exhibited a significant toxic effect in a lethality test of brine shrimp. Furthermore, the pharmacological analysis showed a substantial action of inhibition against the *α*-chymotrypsin and urease enzyme in the alkaloids fraction, prompting us to perform research on phytoconstituents of the plant. As a result of phytochemical work on this plant, four alkaloids were isolated: Bisindigotin (**1**) [11], Candidine (**2**) [12], Isaindigotidione (**3**) [13], and Isaindigotone (**4**) [13], as indicated in Figure 1. To evaluate the structures of alkaloids **1**-**4**, the modern spectroscopy, including the NMR data of 1D and 2D, was used, and their spectral and physical data was in good agreement with those which are previously published for these compounds [11–13]. Despite the fact that the structures of these compounds (**1-4**) have been described earlier in the literature, these compounds were first time isolated from this species. In addition, this research investigates the molecular docking studies of compounds **1-4**, as well as the inhibitory actions of urease and *α*-chymotrypsin, which are not published earlier.

The article "Urease and α-Chymotrypsin Inhibitory Activities and Molecular Docking Studies of Alkaloids Isolated from Medicinal Plant Isatis minima Bunge" was published in 2022. Journal: Evid Based Complement Alternat Med.

A major virulence factor in the pathogenesis was urease (EC 3.5.1.5) that has been proven to be a variety of clinical disorders, posing a risk to agriculture, animal, and human health. Urease is strongly associated with the activation of stones infection and also assists in pathophysiology of hepatic coma, ammonia, urolithiasis, urinary catheter encrustation, pyelonephritis, and hepatic encephalopathy [14, 15]. It is chosen to become the significant source of *Helicobacter pylori* (HP), the diseases referring pathologies. Since during colonization, it permits bacteria to colonize in the stomach at a low pH and hence plays a critical function in development of peptic and gastric ulcers, including cancer [15]. During urea fertilization, maximum urease activity causes substantial economic and environmental concerns in agriculture, since it releases an unusually high amount of ammonia into the atmosphere. That causes damage to the plant, first by restricting them from a vital mineral and next by generating the ammonia concentration which causes toxicity and also rises the pH level in the soil [16, 17].

Urease is a nickel containing metalloenzyme, which catalyzes the hydrolysis of urea into ammonia and carbamic acid, thus resulting in elevation in pH and enabling *H. pylori* to survive in the extreme acidic conditions of stomach [18]. Urease inhibitors, also known as proton pump inhibitors (PPIs), play a vital role in controlling the activity of *H. pylori* by inhibiting the excess ureases secreted [19]. Moreover, a recent study suggests that most of the Proton Pump Inhibitors (PPIs) used in the treatment of stomach ulcers including esomeprazole, omeprazole, rabeprazole, and so on have been risked with severe kidney and liver diseases [20]. In this regard, there is a need of more effective PPIs or urease inhibitors with enhanced biocompatibility and less cytotoxic molecules. The *α*-chymotrypsin inhibitor plays an important role in physiological functions that has been demonstrated in the literature. It also suggests that, in plants' natural defense system, the aforementioned inhibitors are the important components against insect proteinases and also operate by inhibiting the pests [21–23]. As a result, in transgenic plants that produce heterologous inhibitors, such inhibitors have attracted a lot of attention, being possible source of synthetic resistance to pests and pathogens [23]. The plants of tobacco were treated along with gene code of inhibitor serine protease that has been developed for the resistance of insect and pest [24]. In vivo and in vitro, the Bowman–Birk protease inhibitors are often considered as a reliable suppressor agent for tumor [25]. Certain fibrous proteins are decomposed by the association of serine proteases including trypsin and chymotrypsin [26]. The hepatitis C virus causes chronic infection that can cause harm to liver, liver cancer, and cirrhosis. The NS3 protease, also referred to as a chymotrypsin-like serine protease, was identical to the active site of chymotrypsin, which was considered to become a target for anti-HIV medicines and is crucial for replication of the virus [27]. Kunitz-type trypsin inhibitors (KTIs) are widespread in plants [28] and venoms [29], and the first Kunitz inhibitor was isolated from soybean in 1945. Since then, quantities of Kunitz-type inhibitors have been characterized from different species varying from plants to animals [30], and animal-derived KTIs have obtained much focus in decades. Due to the wide distribution, in addition to inhibitory activity, KTIs have been utilized in many other situations. These include potent anticarcinogenic activity in the animal-mimetic environment [31] through blocking urokinase-type plasminogen activator to suppress ovarian cancer cell invasion [32]. In order to discover something new, the identification of an effective inhibitors of *α*-chymotrypsin was the top priority for pharmaceutical development.

The article "Urease and α-Chymotrypsin Inhibitory Activities and Molecular Docking Studies of Alkaloids Isolated from Medicinal Plant Isatis minima Bunge" was published in 2022. Journal: Evid Based Complement Alternat Med.

In the current study, we have described the urease and *α*-chymotrypsin inhibitory activities of the alkaloids (**1-4**) which were isolated for the first time from *Isatis minima* Bunge; however, the structures of the compounds were published previously [11–13] not their urease, *α*-chymotrypsin activities, and molecular docking analysis.

## 2. Materials and Methods

### 2.1. Chemicals and Enzymes

Solvents such as dichloromethane (CH_2_Cl_2_), methanol (MeOH), diethyl ether (Et_2_O), and ethanol (EtOH) were purchased from Aldrich (China). Urease and *α*-chymotrypsin were purchased from Sigma-Aldrich (China); all the other solvents/reagents used were of analytical grade.

### 2.2. Plant Collection

The green whole plant of *Isatis minima* Bunge was harvested in Quetta, Baluchistan, in April 2009 and was authenticated by the plant taxonomist Prof. Dr. Rassol B. Tareen, Department of Botany, University of Baluchistan. A voucher specimen (BUB-321) was preserved on a sheet of herbarium at the University of Baluchistan, Department of Botany in Quetta, Pakistan.

### 2.3. Plant Extraction and Isolation

The whole-plant *Isatis minima* Bunge was shade-dried at room temperature and then 8 kg plant was crushed and filtered three times with 20 L EtOH for 96 hours. The vacuum oven, which was used to evaporate the ethanolic extract, yielded (110 g) a residue that was dark greenish and segregated into the water and EtOAc. The 10% NH_4_OH was used to basified fraction of water; then CH_2_Cl_2_ was employed for extraction. The CH_2_Cl_2_ fraction (17 g) was subjected to column chromatography eluting with *n*-hexane-EtOAc in increasing order of polarity to obtain subfractions. These subfractions rechromatographed over silica gel using *n*-hexane: EtOAc as solvent systems. These fractions were afforded four compounds at different polarity of solvent system as follows: compound **1** (14 mg; solvent system 7 : 3), compound **2** (18 mg; solvent system 8 : 2), compound **3** (17 mg; solvent system 5 : 5), and compound **4** (19 mg; solvent system 6 : 4).

### 2.4. In Vitro Urease Inhibition Assay

In 96-well plates, reaction mixtures containing 25 *μ*L solution of enzyme (urease from *Bacillus pasteurii* and Jack bean) were 30 minutes incubated with 5 *μ*L tested compounds at the temperature of 30°C for 15 minutes, followed by buffers of 55 *μ*L with urea of 100 mM was passed through the process of incubation for 15 minutes. Finally, the technique of indophenol, published by Weatherburn, was accessed for maximum activity of urease through observing the formation of ammonia [17]. Each well received 70 *μ*L of alkali reagent (0.1 percent active chloride NaOCl and 0.5 percent w/v NaOH) and 45 *μ*L of phenol reagent (0.005 percent w/v sodium nitroprusside and 1 percent w/v phenol). The maximum absorbance was recorded at a range of 630 nm by employing a microplate reader molecular device (USA) after 50 minutes. In a final volume of 200 *μ*L, all reactions were repeated in triplicate. The molecular device (USA) program SoftMax Pro was used to process the results. All the experiments were carried out in a potassium phosphate buffer with a pH of 6.8 (1 mM EDTA, 0.01 MK_2_HPO_4_.3H_2_O, and 0.01 M LiCl and HCl were employed to change pH). The equation 100 −(OD_testwell_/OD_control_) × 100 was used to calculate percentage inhibitions. For the standard urease inhibitor, the thiourea was employed. Both ureases were purchased as 99.9% pure from Sigma-Aldrich.

The article "Urease and α-Chymotrypsin Inhibitory Activities and Molecular Docking Studies of Alkaloids Isolated from Medicinal Plant Isatis minima Bunge" was published in 2022. Journal: Evid Based Complement Alternat Med.

### 2.5. In Vitro Chymotrypsin Inhibition Assay

The compounds **1-4** showed inhibition action towards chymotrypsin was evaluated via the Cannel et al. technique [33]. Enzyme chymotrypsin (9 units/mL of 50 mM Tris-HCl buffer pH 7.6; Sigma-Aldrich Chemicals (St. Louis, Mo, USA) were preincubated by different concentrations of the examine compounds at 25°C, for 20 minutes, respectively. Furthermore, 100 *μ*L of substrate solution (1 mg/mL of 50 mM Tris-HCl buffer pH 7.6, *N*-succinyl-phenylalanine-*p*-nitroanilide) is integrated on setting the reaction of enzyme. The liberated *p*-nitroaniline showed absorbance at the range of 410 nm that was constantly measured; up to a substantial colour shift was observed. In reaction mixture, the ultimate concentration of DMSO was 7%.

### 2.6. Determination of IC_50_ Values

The software EZ-Fit Enzyme kinetics (Perrella Scientific Inc., Amherst, USA) was used for measuring the values of IC50 of compounds (1-4) at different concentration.

### 2.7. Molecular Docking

An effective molecular docking approach was used for analyzing the interaction between the target protein and inhibitor molecule [34]. The MOE-Dock software was used to investigate the interaction of binding of such compounds within the active sites of *α*-chymotrypsin, *Bacillus pasteurii* urease, and Jack bean urease. The crystal structures of *α*-chymotrypsin and *Bacillus pasteurii* urease were downloaded with PDB id: 4q2k and 1ubp, respectively, while the Protein Databank (PDB) was used to obtain the Jack bean urease (4 h 9 m). Prior to molecular docking, the program molecular operating environment (http://www.chemcomp.com) was used for eliminating the molecules of water and ions from the acquired structure of crystal to add the atoms of hydrogen into structures of proteins through (3D) protonation and then, MOE's default parameters (gradient: 0.05, force field: Amber99) was used for achieving minimization of energy.

Molecular operating environment program was employed to build the structures of alkaloids **1-4**, and the reduction of energy was observed by operating the default parameters of MOE. The default Molecular Operating Environment software settings permitted *Bacillus pasteurii* urease, *α*-chymotrypsin, and Jack bean urease to dock the compounds (i.e., Rescoring: London dG; Placement: Triangle Matcher). Hence, ten different conformations were synthesized for each ligand. For further investigation, the top-ranking conformation was utilized for each compound. PyMOL software was used to assess the ideal poses with arene-arene, polar, pi-H interactions, and H-pi after molecular docking.

## 3. Results and Discussion

Medicinal plants are used for the treatment of different infections. World Health Organization reports that various plant fractions and their dynamic constituents are utilized as traditional medicines by 80% of the world population [35–39]. Therefore, keeping in mind the importance of medicinal plants, the ethanolic extract of *Isatis minima* Bunge was partitioned between EtOAc and water. Alkaloids liberated from the aqueous fraction with 10% NH_4_OH were extracted out with CH_2_Cl_2_. Column chromatography of CH_2_Cl_2_ fraction provided the alkaloids **1-4**. As the structures of these compounds (**1**–**4**) are known, their physical and spectral data is already reported in literature [11–13]. Herein, in this article, we are reporting docking and enzyme inhibition studies for compounds **1**–**4** for the first time.

The article "Urease and α-Chymotrypsin Inhibitory Activities and Molecular Docking Studies of Alkaloids Isolated from Medicinal Plant Isatis minima Bunge" was published in 2022. Journal: Evid Based Complement Alternat Med.

### 3.1. Urease Inhibitory Activities of Alkaloids **1**–**4**

The alkaloids **1-4** were investigated in order to show the urease inhibition activities as revealed in Table 1. Isaindigotidione (**3**) and Isaindigotone (**4**) displayed potent inhibitory potential against the enzyme with IC_50_ values 34.03 ± 0.07, 26.13 ± 0.08 and 29.03 ± 0.04, 20.04 ± 0.09 *μ*M against *Bacillus pasteurii* and Jack bean urease, respectively. Compounds 1 and 2 showed significant inhibitory activity against both ureases (Table 1). The standard inhibitor of *Bacillus pasteurii* and Jack bean urease (thiourea) had IC_50_ values of 14.03 ± 0.08 and 18.04 ± 0.01 *μ*M, respectively.

### 3.2. *α*-Chymotrypsin Inhibitory Activities of Alkaloids **1**–**4**

The alkaloids **1-4** were evaluated for the inhibition activities of *α*-chymotrypsin as shown in Table 1. Compounds 3 and 4 inhibited *α*-chymotrypsin enzyme in a concentration-dependent manner with IC_50_ values 16.09 ± 0.07 and 22.01 ± 0.06 *μ*M, respectively, whereas the positive control, chymostatin, had an IC_50_ value 7.08 ± 0.07 *μ*M (Table 1). Therefore, both the isolated compounds 3 and 4 have significant potential to bind and inhibit *α*-chymotrypsin enzyme. On the other hand, Bisindigotin (**1**) and Candidine (**2**) displayed moderate inhibitory potential against *α*-chymotrypsin (Table 1).

### 3.3. Structure Activity Relationship (SAR) Studies of Alkaloids 1-4

The results (as given in Table 1) showed that compounds containing more methoxy, carbonyl, and hydroxyl groups were the powerful inhibitors of the two enzymes. Compound **3** was extremely efficient as compared to other compounds because it contains more methoxy, carbonyl, and hydroxyl groups and also exhibiting IC_50_ values 20.04 ± 0.09 *μ*M and 29.03 ± 0.04 *μ*M against *Bacillus pasteurii* urease and Jack bean, respectively. Furthermore, it exhibited strong inhibition capability with IC_50_ values of 16.09 ± 0.07 *μ*M against *α*-chymotrypsin. Compound **4** exhibited the second maximum inhibition with one carbonyl, one hydroxyl, and two methoxy groups while compound **2** demonstrated the minimum inhibition against the two enzymes in this series, exhibiting small number of hydroxyls, carbonyl, and methoxy group. It revealed that inhibitory action slightly increases with increasing numbers of methoxy, hydroxyl, and carbonyl groups. This is because of the chelation of such groups with the enzyme active site, which increases the inhibition activity of these compounds. Apparently, a number of concerns about the action mode of such ligands remain unanswered, and the solutions to these issues will be critical in the establishment of future decades of these inhibitors. As a result, we will analyze different derivatives of compounds **1-4** to investigate in vitro against *α*-chymotrypsin and urease using molecular dynamics simulations, STD NMR, and kinetics investigations in order to determine the exact inhibition mechanism of these compounds.

The article "Urease and α-Chymotrypsin Inhibitory Activities and Molecular Docking Studies of Alkaloids Isolated from Medicinal Plant Isatis minima Bunge" was published in 2022. Journal: Evid Based Complement Alternat Med.

### 3.4. Docking Analysis of Jack Bean Urease Enzyme

The binding mechanism of alkaloids **1-4** was investigated using molecular docking. According to the molecular docking experiments, Table 2 showed all the compounds that have high level of conformations and tightly fitted into the enzyme Jack bean urease active site (Arg 439, Ala 440, Thr 441, KCX 490, CME 592, His 593, Arg 609, Asp 633, Gln 635, and Met 637). As a result, docking conformation analysis of all the compounds demonstrate that compound **3** identified four polar bonds, two H-pi, and one pi-Isaindigotidione (IC_50_ = 29.03 ± 0.04 *μ*M, docking score = − 13.1927) pi linkage with Arg 439, Ala 440, Ala 636, Arg 609, and His 593 of the urease enzymes, respectively. The oxygen atoms of the compound form hydrogen bonds with Arg 439, Ala 636, and Arg 609, as illustrated in Figure 2. The Ala 440 residues of the target protein formed a polar bond with the amine group of a nitrogen atom, whereas His 593 formed Hi-pi and arene-arene interactions with the compound 6-ring moiety. An electron flow in the compound was produced because of the presence of hydroxyl and methyl groups, which act as an electron-donating group and electron-accepting group like carbonyl oxygen, forming the more potent, polarizable, and active compound, which may demonstrate the strong inhibitory action.

### 3.5. Docking Analysis of *Bacillus pasteurii* Urease Enzyme

In this analysis, most active compound **3** showed the maximum docking score (−8.6876) along with the inhibitory action (IC_50_ = 20.04 ± 0.09). The coupling compound **3** with the urease enzyme in an appropriate way via one arene-arene and three hydrogen bond linkage in Figure 3; Table 3. The –NH and the oxygen of the carbonyl groups of a compound form the hydrogen bonding interaction in the residue His 323, whereas His 222 established a polar interaction with the hydroxyl group of a compound. The exitance of electron-accepting groups, such as oxygen atoms of carbonyl group and electron-donating groups, such as -OH group, showed strong inhibitory potential of the compounds.

The article "Urease and α-Chymotrypsin Inhibitory Activities and Molecular Docking Studies of Alkaloids Isolated from Medicinal Plant Isatis minima Bunge" was published in 2022. Journal: Evid Based Complement Alternat Med.

### 3.6. Docking Analysis of *α*-Chymotrypsin

For most active compound **3** (IC_50_ = 16.09 ± 0.07, docking score = − 7.6647), the amino acid residues Asp102, Met 192, Ser195, and Gly 216 created a network of hydrogen bonds with the proton of a hydroxyl group and oxygen atoms of a methoxy group of a compound as seen in Figure 4. The existence of electronegative, electron-donating groups as well as the electron cloud system of a compound determines the inhibitory effect of a compounds.  Table 4 mentioned the interaction reports of the remaining compounds.

Overall, the significant correlation between the biological activities and docking scores of such compounds was investigated with Jack bean urease enzyme, *bacillus pasteurii* urease enzyme, and *α*-chymotrypsin, respectively (Figures 5(a)–5(c)).

Experimental as well as docking studies have proven that the compounds (**1**–**4**) have shown dual inhibiting properties for enzymes unease and *α*-chymotrypsin because compounds **1**–**4** have common functional groups (carbonyl, hydroxyl, and methoxy moieties), which bind to the active site of both the enzymes urease and *α*-chymotrypsin. The data reflect that compound **3** and compound **4** have potent dual inhibitors role, have significance IC_50_ values, and also confirm by docking studies against the ureases and *α*-chymotrypsin. The docking studies of compounds **3** and **4** against the respective enzymes have predicted strong binding sites to interact with specific residues in enzymes active sites, showing strong inhibitory potential of the compounds against respective enzymes, as fact provided in the docking studies of the compounds.

The body of evidence presented in the review by Modolo et al. clearly demonstrates the great potential of plant extracts and their secondary metabolites to negatively affect the activity of ureases. Different classes of natural products like alkaloids, cardiac glycosides, saponins, polyphenolics, and flavonoids were reported for their urease activities [40]. Similarly, antiurease, *α*-glucosidase, and antilipoxygenase activity is reported in the literature for crude alkaloids from fruit, bark, leaves, and root of *Zanthoxylum armatum* [41]. Alkaloids isolated from different plants were also investigated for their *α*-chymotrypsin inhibitory potential [42–44]. The above reported data support the urease *α*-chymotrypsin inhibitory activities of our alkaloids **1**–**4**.

The article "Urease and α-Chymotrypsin Inhibitory Activities and Molecular Docking Studies of Alkaloids Isolated from Medicinal Plant Isatis minima Bunge" was published in 2022. Journal: Evid Based Complement Alternat Med.

## 4. Conclusion

In conclusion, our search for urease and protease inhibitory constituents from *Isatis minima* Bunge has resulted in the isolation of alkaloids **1**–**4**, as potential agents in the treatment urease- and *α*-chymotrypsin-associated complications. However, a further in vivo study would help in providing further insight into the pharmacological properties of these lead compounds. The molecular docking studies confirmed that these alkaloids isolated from *Isatis minima* were competitive inhibitors. A chemical scaffold for such types of compounds with potent results leads to novel drugs.

## Figures and Tables

**Figure 1:** Structure of compounds **1**–**4**.

**Figure 2:** Docking orientation of compound **3** with the Jack bean urease enzyme active site.

**Figure 3:** Docking orientation of compound **3** with the *Bacillus pasteurii* urease enzyme active site.

**Figure 4:** Docking orientation of compound 3 on active site of *α-*chymotrypsin.

**Figure 5:** Activity of docking and IC_50_ values graph prediction for (a) Jack bean urease, (b) *Bacillus pasteurii* urease enzyme, and (c) *α*-chymotrypsin enzyme.

**Table 1:** In vitro inhibition of urease and *α*-chymotrypsin by alkaloids **1**–**4**.

Compounds	Urease IC_50_ ± SEM^a)^ [*μ*M]		*α*-Chymotrypsin
	(*Bacillus pasteurii* urease)	(Jack bean urease)	
			IC_50_ ± SEM^a)^ (*μ*M)
Bisindigotin	42.04 ± 0.07	58.15 ± 0.02	34.01 ± 0.07
Candidine	46.12 ± 0.05	68.21 ± 0.08	44.07 ± 0.04
Isaindigotidione	20.04 ± 0.09	29.03 ± 0.04	16.09 ± 0.07
Isaindigotone	26.13 ± 0.08	34.03 ± 0.07	22.01 ± 0.06
Thiourea^b^	14.03 ± 0.08	18.04 ± 0.01	—
Chymostatin^c^	—	—	9.01 ± 0.02

^a^Standard mean error of five determinations; ^b^ positive control used in urease inhibiting assay; and ^c^ positive control used in chymotrypsin assays.

**Table 2:** Potential interaction research and docking score of dock conformations towards Jack bean urease.

S. no.	Docking scores	Ligand		Receptor				Interaction	Distance	*E* (kcal/mol)
**1**	−10.825	**C**	30	SG	CME	592	(A)	H-donor	3.12	−0.2
		C	32	O	GLN	635	(A)	H-donor	3.67	−0.1
		C	34	SG	CME	592	(A)	H-donor	3.11	−0.2
		C	36	O	ARG	439	(A)	H-donor	2.81	−0.1
		N	45	O	ALA	436	(A)	H-donor	2.86	−2.9
		N	40	CB	ARG	439	(A)	H-acceptor	3.21	−0.3
		N	40	CB	ALA	440	(A)	H-acceptor	3.95	−0.1
		NI	902	OQ2	KCX	490	(A)	Metal	1.99	−6.3
		NI	902	ND1	HIS	519	(A)	Metal	2.14	−4.5
		NI	902	OQ1	KCX	490	(A)	Ionic	3.39	−2.3
		NI	902	OQ2	KCX	490	(A)	Ionic	1.99	−16.4
		5-Ring		NH2	ARG	439	(A)	Pi-cation	3.91	−0.6
		5-Ring		CB	ALA	440	(A)	Pi-H	3.82	−0.2
**2**	−8.9541	C	22	O	ALA	636	(A)	H-donor	3.5	−0.1
		O	1	NH1	ARG	609	(A)	H-acceptor	3.77	−0.6
		O	32	CA	HIS	593	(A)	H-acceptor	4.3	−0.1
		6-Ring		5-Ring	HIS	593	(A)	Pi-Pi	3.94	0
**3**	−13.1927	O	16	CA	ALA	440	(A)	H-acceptor	3.49	−0.5
		O	16	CB	ALA	636	(A)	H-acceptor	4.03	−0.2
		O	30	NH2	ARG	439	(A)	H-acceptor	3.09	−3.7
		O	44	NH2	ARG	609	(A)	H-acceptor	3.13	−2.5
		C	24	5-Ring	HIS	593	(A)	H-Pi	3.89	−0.1
		C	45	5-Ring	HIS	593	(A)	H-Pi	4.33	−0.1
		6-ring		5-Ring	HIS	593	(A)	Pi-Pi	3.95	0
**4**	−11.2329	C	29	O	ARG	439	(A)	H-donor	3.86	−0.1
		O	20	NH2	ARG	439	(A)	H-acceptor	2.87	−5.8
		O	35	NE2	HIS	492	(A)	H-acceptor	3	−1.7
		O	35	CE1	HIS	519	(A)	H-acceptor	2.88	−0.1
		O	35	NI	NI	902	(A)	Metal	2.71	−1.7
		NI	902	OQ2	KCX	490	(A)	Metal	1.99	−6.3
		NI	902	ND1	HIS	519	(A)	Metal	2.14	−4.5
		NI	901	OQ1	KCX	490	(A)	Metal	2.08	−5.2
		NI	901	OD1	ASP	633	(A)	Metal	2.12	−4.2
		NI	901	OQ2	KCX	490	(A)	Ionic	3.39	−2.4
		NI	901	OD1	ASP	633	(A)	Ionic	2.12	−14.1
		6-Ring		CZ	CME	592	(A)	Pi-H	3.73	−0.3

The article "Urease and α-Chymotrypsin Inhibitory Activities and Molecular Docking Studies of Alkaloids Isolated from Medicinal Plant Isatis minima Bunge" was published in 2022. Journal: Evid Based Complement Alternat Med.

**Table 3:** Potential interaction research and docking score of dock conformations towards *Bacillus pasteurii* urease.

S. no.	Docking scores	Ligand	Receptor				Interaction	Distance	*E* (kcal/mol)
**1**	−7.1082	C 30	6-Ring	TRP	225	(C)	H-Pi	4.08	−0.1
		6-Ring	CA	GLY	167	(C)	Pi-H	4.9	−0.1
		5-Ring	CB	HIS	324	(C)	Pi-H	4.06	−1.4
		6-Ring	CB	HIS	324	(C)	Pi-H	4.79	−0.3
		5-Ring	CD2	HIS	324	(C)	Pi-H	4.04	−0.3
		6-Ring	5-Ring	HIS	324	(C)	Pi-Pi	3.8	0
**2**	−5.9783	C 24	SG	CYS	322	(C)	H-donor	3.45	−0.1
		O 32	NZ	LYS	169	(C)	H-acceptor	3.13	−1.9
		C 40	5-Ring	HIS	324	(C)	H-Pi	3.98	−0.3
		5-Ring	CD	LYS	169	(C)	Pi-H	4.13	−0.4
**3**	−8.6876	N 11	OD2	HIS	323	(C)	H-donor	2.75	−3.6
		O 42	N	HIS	323	(C)	H-donor	2.66	−1.7
		O 30	NZ	HIS	222	(C)	H-acceptor	2.87	−2.5
**4**	−7.8349	C 1	OD1	ASP	224	(C)	H-donor	3.34	−0.2
		C 41	OD1	ASP	332	(C)	H-donor	3.58	−0.2

**Table 4:** Potential interaction research and docking score of dock conformation towards *α*-chymotrypsin enzyme.

S. no.	Docking scores	Ligand	Receptor				Interaction	Distance	*E* (kcal/mol)
**1**	−7.6644	O 44	CA	MET	192	(A)	H-acceptor	3.33	−0.2
		5-Ring	CB	HIS	57	(A)	Pi-H	4.58	−0.4
		6-Ring	CB	HIS	57	(A)	Pi-H	4.66	−0.4
		6-Ring	NZ	LYS	93	(A)	Pi-cation	3.53	−0.2
		5-Ring	CG	MET	192	(A)	Pi-H	4	−0.4
		5-Ring	CA	TRP	215	(A)	Pi-H	4.75	−0.2
		6-Ring	CA	TRP	215	(A)	Pi-H	4.35	−0.3
		6-Ring	N	GLY	216	(A)	Pi-H	3.96	−0.3
**2**	−7.0753	O 1	CA	MET	192	(A)	H-acceptor	3.34	−0.5
		O 32	NZ	LYS	93	(A)	H-acceptor	3.2	−0.7
		5-Ring	CB	HIS	57	(A)	Pi-H	4.34	−0.2
		6-Ring	CB	HIS	57	(A)	Pi-H	4.74	−0.2
		6-Ring	CE	LYS	93	(A)	Pi-H	4.31	−0.3
		6-Ring	CG	MET	192	(A)	Pi-H	4.99	−0.3
		5-Ring	OG	SER	195	(A)	Pi-H	3.7	−0.2
		6-Ring	CA	TRP	215	(A)	Pi-H	4.92	−0.2
		6-Ring	CA	TRP	215	(A)	Pi-H	4.01	−0.6
		6-Ring	CB	TRP	215	(A)	Pi-H	4.08	−0.4
		6-Ring	N	GLY	216	(A)	Pi-H	4.17	−0.2
**3**	−7.6647	O 44	O	SER	195	(A)	H-donor	3.9	−0.4
		C 45	SD	MET	192	(A)	H-donor	4.12	−0.3
		O 1	O	ASP	102	(A)	H-donor	3.73	−0.4
		O 16	NH	GLY	216	(A)	H-acceptor	3.39	−0.1
		O 30	NH	MET	192	(A)	Pi-H	4.44	−0.1
		6-Ring	CG	MET	192	(A)	Pi-H	3.73	−0.3
		6-Ring	CA	TRP	215	(A)	Pi-H	4.61	-0.2
**4**	−7.5727	O 20	NZ	LYS	175	(A)	H-acceptor	2.94	−6.4
		O 35	CA	MET	192	(A)	H-acceptor	3.62	−0.2
		O 35	CG	MET	192	(A)	H-acceptor	3.99	−0.1
		6-Ring	CG	MET	192	(A)	Pi-H	4.39	−0.2
		6-Ring	CA	TRP	215	(A)	Pi-H	4.15	−0.5
		6-Ring	N	GLY	216	(A)	Pi-H	4.41	−0.1

The article "Urease and α-Chymotrypsin Inhibitory Activities and Molecular Docking Studies of Alkaloids Isolated from Medicinal Plant Isatis minima Bunge" was published in 2022. Journal: Evid Based Complement Alternat Med.

## Data Availability

All the available data are incorporated in the paper.
